# Observation of Clinical Efficacy of Anisodamine and Chlorpromazine in the Treatment of Intractable Hiccup after Stroke

**DOI:** 10.1155/2022/6563193

**Published:** 2022-07-11

**Authors:** Jing Wang, Qinghua Zhu, Shuyan Zhang, Lisha Wen, Li Wang

**Affiliations:** Department of Neurology, Affiliated Hospital of Hebei University of Engineering, Handan, 056002 Hebei, China

## Abstract

**Objective:**

This study is aimed at investigating the clinical efficacy of anisodamine combined with chlorpromazine on intractable hiccups after stroke.

**Methods:**

150 patients admitted to Affiliated Hospital of the Hebei University of Engineering from 2017 to 2021 were selected as the research objects, all of which received the computed tomography (CT) examination. During CT examination, intelligent algorithms were used to segment the images. An unsupervised multilayer image threshold segmentation algorithm was proposed by using Kullback-Leibler (K-L) divergence and the modified particle swarm optimization (MPSO) algorithm. All patients were divided into three groups, with each group of 50 patients. Patients in the control group (group A) took the calcium tablets, vitamin C tablets, and vitamin B1 tablets orally. Patients in the control group (group B) received the acupoint injection of anisodamine, and those in the observation group (group C) received the acupoint injection of anisodamine combined with chlorpromazine. The therapeutic effect and patient satisfaction of the three groups were compared.

**Results:**

The two-dimensional (2D) K-L divergence was applied for the multilayer segmentation of images, which was helpful to obtain accurate images. The MPSO algorithm was adopted to reduce the computational complexity. The total efficiency of group C was 98%, that of group B was 56%, and that of group A was 22%. The total efficiency and satisfaction rate of group C were signally better than those of group A and group B (*P* < 0.05).

**Conclusion:**

The combination of 2D K-L divergence and MPSO algorithm could improve the accuracy of multilayer image segmentation and CT imaging. Acupoint injection of anisodamine combined with chlorpromazine had better efficacy than the injection of anisodamine alone for the treatment of intractable hiccups after stroke, with high safety and clinical promotion value.

## 1. Introduction

Stroke refers to a bunch of conditions associated with blockage or bursting of the artery that imparts blood to the brain. It is the second leading cause of death around the globe, with 15 million new cases, around 5 million permanent disabilities, and 5 million deaths each year. In China, the situation is quite alarming with approximately 2.5 million new cases, accompanied by a 75% disability rate which poses a high risk to individuals, families, and society regarding their health [1, 2]. With the aging of the population and the continuous development of medical treatment, the mortality of stroke decreases gradually but incidence and complications after stroke increase cautiously. Intractable hiccup is one of the common complications after stroke. Hiccup is a relatively universal physiological phenomenon, especially in stroke patients, which refers the gas in the stomach making a quick and short sound from the throat. The respiratory center of patients is directly or indirectly affected by the lesions, and the duration is prolonged. If a hiccup occurs for more than 48 h, it is called an intractable hiccup [5, 6]. Clinically, it can be caused by various factors like gastrointestinal dysfunction, electrolyte disorder, mental factors, and primary or secondary brain stem damage. If it is not well controlled, it will lead to some unexpected events and bring serious threats to the physical and mental health of patients [3, 4]. Stroke is often accompanied by intermittent and recurrent hiccups sometimes followed by vomiting, reflux, aspiration, and other aggravating conditions which not only affect patients' sleep but also make them in a poor mood [7–9]. Stroke patients with dry heat, hyperactivity of liver-yang, qi stagnation and phlegm obstruction, and deficiency of liver-yin and kidney-yin can cause the internal wind to multiply the lung and stomach, which results in gastric qi trapping on the phlegm and moving the diaphragm, thus causing hiccups [10–13]. According to some research, chlorpromazine is injected into the bilateral Neiguan acupoint for the treatment of intractable hiccups, which has good effects. Besides, chlorpromazine can block *α* adrenergic receptors of the ascending activating system of the reticular structure, which is used for the treatment of intractable hiccups [14]. Due to this side effect, chlorpromazine cannot be utilized solely for the treatment of intractable hiccups. Anisodamine is used for the treatment of vascular spasms and embolism associated with circulation disorders, relieving the colic caused by the gastrointestinal tract, biliary tract, and other spasms. According to the pharmacodynamics of anisodamine, it is helpful in overcoming the side effects of chlorpromazine by improving microcirculation and relieving vasospasm, with a theoretical basis for the treatment of intractable hiccups. It can reduce saliva secretion, with a certain synergistic effect [15].

Various medical imaging techniques have been employed to obtain detailed images of many interior parts of the body for the diagnosis of many diseases. Advancement in computer information systems, intelligent computing has been applied more and more widely in computed tomography/magnetic resonance imaging image processing (CT/MRI) [16]. Image segmentation is also a key step in medical image processing. Based on computer vision technology, the original image can be transformed into an abstract form to obtain a high level of comprehension [17]. Over the years, many types of segmentation algorithms are proposed, and each has certain pros and cons. There also exists diversity in image segmentation methods, including the neural network method, contour extraction method, image segmentation method, and threshold segmentation method. The solid theoretical foundation is widely used in various image segmentations. With the emergence of multitarget tracking and optimization, the selection of two parts of the image cannot meet the needs of identifying information. Multiple thresholds are used to segment the image into multiple targets, which is conducive to the calculation of segmentation and reducing the complexity [18–20]. Among diverse image segmentation algorithms, the particle swarm optimization (PSO) algorithm is preferred due to its simplicity, having multiple thresholds, and being widely utilized for image segmentation in recent years. It is suitable for nonlinear optimization problems in multidimensional space, with few parameters, simple structure, and easy implementation [21]. In mathematical probability statistics, divergence refers to a function that measures similarity between two distributions. Kullback-Leibler (K-L) divergence is a kind of relative entropy to measure the theoretical distance between the information distribution *P* and *Q*. K-L can be understood that *M* is replaced by *N*, namely, the expectation of information content changes. The fewer information changes are, the smaller the divergence value is [22].

The patients with intractable hiccups after stroke undergo a CT scan; then an unsupervised multilayer image threshold segmentation algorithm with the combined effect of two-dimensional (2D) K-L divergence and MPSO was proposed to perform the multiple segmentation of CT images. The clinical efficacy of anisodamine combined with chlorpromazine had been investigated by injecting it at bilateral Neiguan acupoint in patients [23, 24]. The intelligent algorithm was introduced into CT imaging to enhance the clarity of images, which was conducive to the diagnosis of patients' diseases. The accuracy of treatment was improved, and it provided a reliable theoretical basis for clinical treatment.

## 2. Materials and Methods

### 2.1. K-L Divergence

In mathematical probability statistics, divergence refers to a function that measures similarity between two distributions. K-L belongs to the measurement of the differences between *M* and *N* whereas *M* and *N* are asymmetric, where *N* represents the estimation of *M*, and *M* represents the real distribution of data. Consequently, divergence is estimating the loss of *M* information with *N*.

*N* : *x*⟶[0, 1] distribution, *α* ∈ [0, 1) ∪ (1, ∞), and *M* : *x*⟶[0, 1] distribution, and the equation is expressed as shown in Equation (1).

(1) $$\begin{array}{c} W_{\alpha }\left(M\left\|N\right.\right)=\log\left[\underset{\text{x}}{\sum }{\frac{M\left(x\right)\alpha }{N\left(\text{x}\right)\alpha -1}}^{1/\alpha ‐1}\right]. \end{array}$$

In Equation (1), *W*_*α*_(*M*‖*N*) represented the distance measurement between the two distributions *M* and *N*, also known as the Renyi divergence. The similarity between *M* and *N* reduces the value of Renyi divergence. The more similar *M* and *N* are, the smaller the value *W*_*α*_(*M*‖*N*) is.

If *α*⟶1, the limiting value Equation (2) of Renyi divergence is like Equation (3).

(2) $$\begin{array}{c} W_{1}\left(M\left\|N\right.\right)=\lim_{\alpha ⟶1}W_{\alpha }\left(M\left\|N\right.\right), \end{array}$$

(3) $$\begin{array}{c} W\left(M\left\|N\right.\right)=\underset{\text{x}}{\sum }p\left(x\right)\log\frac{M\left(x\right)}{N\left(\text{x}\right)}. \end{array}$$

Equation (3) requires that *M* and *N* have the same dimension, and Equation (4) is obtained.

(4) $$\begin{array}{c} \underset{\text{xi}}{\sum }p\left(xi\right)=\underset{xi}{\sum }q\left(xi\right). \end{array}$$

In the image segmentation, *M* expresses the original images, and *N* expresses the corresponding segmentation results.

### 2.2. The Relationship between Divergence and Image Segmentation

The task of image segmentation is to make the segmented image just like the original one. The divergence is employed to calculate varying degree of the information before and after image segmentation so that we have an idea about information loss during segmentation. A smaller divergence value will lead to a better segmentation effect. *F*(*x*, *y*) ∈ (0, 1, 2, ⋯, 255) represents the images before the segmentation, and the segmented image is represented by *g*(*x*, *y*).

(5) $$\begin{array}{c} \text{g}\left(x,y\right)=\left\{\begin{array}{c} {\text{s}}_{1}f\left(x,y\right)\leq \text{t},\\ s_{2}f\left(x,y\right)>\text{t}. \end{array}\right. \end{array}$$

In Equation (5), *S*_1_ and *S*_2_ represent the Gray values of the background and foreground after image segmentation.

For the divergence value of images *f* and *g*, Equation (6) is used to illustrate the advantages and disadvantages of segmented images.

(6) $$\begin{array}{c} W\left(f\left\|g\right.\right)=\overset{n}{\underset{i=0}{\sum }}f_{i}\log\frac{f_{i}}{g_{i}}+\overset{A}{\underset{i=\text{n}+1}{\sum }}f_{i}\log\frac{f_{i}}{g_{i}}. \end{array}$$

In Equation (6), *A* presents the maximum Gray value of the image, and *f*_*i*_ and *g*_*j*_ present the number of pixels of Gray value *i* before and after image segmentation. The smaller the change between segmented and nonsegmented images, the better will be segmentation effect is. Hence, segmentation is finding the optimal threshold *T*∗ to minimize the value of the objective function. Equation (7) shows the threshold function.

(7) $$\begin{array}{c} T*=\arg\min tW\left(f\left\|g\right.\right). \end{array}$$

The image values before and after segmentation meet the conditions of Equations (8)–(10).

(8) $$\begin{array}{c} \text{num}\left(f_{j}\right)=\text{num}\left(g_{j}\right), \end{array}$$

(9) $$\begin{array}{c} \overset{n}{\underset{i=0}{\sum }}f_{i}=\overset{\text{n}}{\underset{i=0}{\sum }}v1, \end{array}$$

(10) $$\begin{array}{c} \overset{A}{\underset{i=n+1}{\sum }}f_{i}=\overset{\text{A}}{\underset{i=n+1}{\sum }}v2. \end{array}$$

The number of pixels before and after image segmentation is the same. The sum of Gray values of the segmented region remains unchanged after segmentation.

### 2.3. Description of Particle Swarm Optimization

Particle swarm optimization (PSO) is a simplified model established by using swarm intelligence. The algorithm is based on the observation of animal cluster activity behaviours. Then, by using the information sharing of the particles in the group, the movement of the whole group can evolve from disorder to order in the problem-solving space. Finally, the optimal solution can be obtained. PSO is an iterative algorithm. Compared with the genetic algorithm, PSO is more simple and easier to implement, and it does not have many parameters to adjust, which can be applied to the optimization of nonlinear functions in the multidimensional space.

In the N-dimensional space, there are *R* particles, and each particle needs to have a rate and position. Equations (11) and (12) show how the rate and position of the *j*-th class of the *i*-th particle are calculated.

(11) $$\begin{array}{c} {\text{v}}_{ij}\left(n+1\right)=w\times v_{ij}\left(n\right)+c_{1}\times {\mathrm{rand}}_{1}\times \left({pBest}_{j}\left(n\right)-x_{ij}\left(n\right)\right)+C_{2}\times {\mathrm{rand}}_{2}\times \left(g{\text{Best}}_{j}\left(n\right)-x_{ij}\left(n\right)\right), \end{array}$$

(12) $$\begin{array}{c} {\text{x}}_{ij}\left(\text{n}+1\right)=x_{ij}\left(n\right)+v_{ij}\left(n+1\right). \end{array}$$

In Equations (11) and (12), *n* represents the current number of iterations, *i* = 1, 2 ⋯ *R* represents the indexes of particles, and *j* = 1, 2 ⋯ *n* represents the dimension of particle space. *C*_1_ and *C*_2_ express the acceleration coefficients, and *W* expresses the degree to which the forward velocity of the particle affects the present velocity.

Equation (13) shows the calculation of the adaptive inertia weight measurement.

(13) $$\begin{array}{c} \text{w}=\frac{w_{\max}-\left(w_{\max}-w_{\min}\right)\text{n}}{K}. \end{array}$$

In Equation (13), *K* presents the total iteration. At this point, *W*_max_ and *W*_min_ have fixed values of 0.9 and 0.4, respectively. Besides, rand_1_ and rand_2_ present the uniformly distributed random numbers within [0, 1], *pg*_*i*_(*n*) presents the global optimal position of the *j*-dimension of particle swarm, and *pi*_*j*_(*n*) presents the optimal individual position of the *j*-dimension of particle *i*.

For the modified particle swarm optimization (MPSO) algorithm, the particle swarm is initialized freely in a suitable space. In this work, an adaptive factor *fα* was adopted, and Equation (11) was modified into Equation (14).

(14) $$\begin{array}{c} x_{ij}\left(n+1\right)=v_{ij}\left(n\right)+f\alpha \times v_{ij}\left(n+1\right)=x_{ij}\left(n\right)+\mathrm{rand}\times \left(1-\frac{t}{K}\right)x_{ij}\left(n+1\right). \end{array}$$

The value of *fα* gradually decreases with the increase of iteration times. Consequently, the value of *fα* is large at the beginning of the iteration. The improved PSO algorithm had a strong ability to continuously detect new regions that replaced the defect of premature convergence, and *fα* could balance the global and local search ability of the algorithm well. Nevertheless, only using adaptive factors could not maintain the excellent merging ability and diversity of the algorithm. In PSO, the global optimal position guides the flight direction of particles, which is conducive to the management of the diversity and convergence of particles. The disturbance range of *g*Best is controlled within [0 max (*x*) − min(*x*)]. Moreover, max(*x*) and min(*x*) represent the difference between the maximum and minimum positions of particles in the iteration. As the number of iterations increases, the value of max(*x*) − min(*x*) decreases gradually. The low disturbance rate makes the algorithm merge gradually, which is helpful to search the optimal value finely. Equation (15) shows the calculation of *g*Best.

(15) $$\begin{array}{c} g{\text{Best}}_{j}=g{\text{Best}}_{j}+ga=g{\text{Best}}_{j}+\left(\max\left(x_{j}\right)-\min\left(x_{j}\right)\right)\times \mathrm{rand}. \end{array}$$

In Algorithm 1, the execution of the MPSO algorithm is described in detail, and it shows the pseudocode of the algorithm.

The combination of MPSO and 2D K-L helps find the optimal threshold in image segmentation, and 2D K-L divergence can be regarded as the fitness function of MPSO to find the optimal threshold in image segmentation.  Figure 1 shows the flow diagram of the multilayer threshold image segmentation algorithm.

## 3. Experiment Environment

MATLAB R2014b was employed in the experiment, and the program was executed on a Celeron 1.8 GHz processor with 10 G memory. Group cognitive parameters, individual cognitive parameters, and particle swarm length were all fixed at 1.43, 0.7, and 20 values, respectively. The convergence performance of threshold algorithms at different layers was evaluated. The number of layers of image segmentation was determined regarding the needs of practical problems, and the convergence performance was analyzed according to the number of iterations in the algorithm.

### 3.1. Research Objects

150 patients admitted to Affiliated Hospital of the Hebei University of Engineering from 2017 to 2021 were selected. All patients were diagnosed with stroke by CT or MRI and complicated with intractable hiccups after onset. The 150 patients were further subcategorized into 82 male patients and 68 female patients, having ages ranging from 37 to 83 years old, approximately (65.96 ± 13.95) years on average. The time duration of the illness was 5-40 days. Among all the research objects, there were 39 cases of cerebral infarction, 35 cases of multiple lumen infarction, 27 cases of lacunar infarction, 14 cases of cerebral hemorrhage, 16 cases of cerebral thrombosis, and 19 cases of subarachnoid hemorrhage. Patients were divided into three groups named control group A, control group B, and observation group C with the help of a randomized, double-blind, and parallel control method which was adopted to averagely divide the patients into three groups.

Patients included in the control group (group A) were given oral calcium tablets, vitamin C tablets, and vitamin B1 tablets.

Patients in the control group (group B) received the acupoint injection of anisodamine alone.

Patients included in the observation group (group C) received the acupoint injection of anisodamine combined with chlorpromazine.

The differences in the disease types, ages, disease conditions, and occurrence time of hiccups among the three groups were not statistically significant (*P* > 0.05). All procedures of this experiment were approved by the ethics committee of Affiliated Hospital of Hebei University of Engineering, and all patients signed the informed consent.

### 3.2. Inclusion Criteria

The inclusion criteria were as follows: (I) patients who had been admitted at Affiliated Hospital of the Hebei University of Engineering for a long period of time, (II) inpatients with clinical treatment (including age, sex, previous medication history, and history of encephalopathy) that were collected in detail, (III) patients who met the diagnostic requirements of various cerebrovascular diseases in the fourth *National Cerebrovascular Disease Academic Conference*, (IV) patients with no other mental diseases, (V) patients with good understanding and communication skills, and (VI) patients who were diagnosed with stroke by MRI or craniocerebral CT with intractable hiccups during hospitalization.

### 3.3. Exclusion Criteria

The exclusion criteria were as follows: (I) patients who did not agree to participate in the experiment, (II) patients with incomplete case data, (III) patients with severe organ dysfunction, (IV) patients with congenital diseases, (V) patients with mental diseases, (VI) patients in lactation and pregnancy, and (VII) patients with malignant tumors.

### 3.4. Methods

Patients in group A were given oral calcium tablets, vitamin C tablets, and vitamin B1 tablets. Patients in group B and group C were injected at the bilateral Zusanli acupoint. During the injection, patients were placed in supine, bent knees, or sitting position, and the Zusanli acupoint was correctly selected and sterilized with 0.5% active iodine. Before treatment, each group of patients was acknowledged with relevant knowledge of Zusanli acupoint and other notes in the treatment process to eliminate the tension between patients and their families. The patient was placed in a comfortable position and was sure to keep warm and be fixed. The syringe was held in the right hand, and the needle was vertically inserted for about 2.5 cm. The method of lifting and thrusting was used to strengthen and control the direction of needle sensation conduction. When there was no blood return on withdrawing the needle, the drug was injected rapidly. Patients in group B were only injected with 10 mg anisodamine, and the needle was injected at a 90-degree angle for 3-4 cm and gently twisted. When patients had a sense of acid swelling, half of the liquid was selected and injected slowly. Meanwhile, the same method was adopted for the side Zusanli acupoint. If it worked, it was repeated within 6 hours. Patients in group C were injected with 10 mg anisodamine and 25 mg chlorpromazine, and the injection method was the same as adopted in the case of group B.

During the operation, the injection part had been fully disinfected through an aseptic technique to prevent any infection. Furthermore, the effect and reactions of patients were attentively noticed. If the patient suffered from needle sickness, bending, and other conditions, the corresponding measures were taken immediately. The personalized treatment procedures were taken according to the different symptoms of the patient.

### 3.5. Evaluation Criteria of Efficacy

Table 1 shows the evaluation criteria of efficacy. Efficiency among patients distributed in various groups can be determined with the help of the following formulas:

(16) $$\begin{array}{c} \text{Efficiency}=\text{cure}+\text{the marked effectiveness}+\text{improvement}. \end{array}$$

According to the abovementioned formula, the efficacy of treatment is not only dependent upon a number of cure cases, but the effective and improved cases' also have a marked impact on total efficiency.

The total efficiency (%) = (the number of marked efficacy cases + the number of effective cases + the number of improvement cases)/the total number of cases × 100%.

Satisfaction rate (%) = (the number of very satisfied cases + the number of satisfied cases)/the total number of cases × 100%.

### 3.6. Statistical Methods

All the data was collected with the help of Excel 2007 and SPSS 21.0. SPSS 21.0 is an advanced analytical tool utilized for data management. Both of this statistical software were employed according to different situations. Mean ± standard deviation ( $\bar{x}$ ± *s*) was used to express that how measurement data conformed to normal distribution while frequency (%) showed how nonconformity count data were expressed, and the data was tested by *χ*^2^ test. Frequency, percentage, mean, and standard deviation were employed to describe general demographic data. The difference was statistically significant *P* < 0.05.

## 4. Results

### 4.1. Comparison of General Data

According to Table 2, in group A, there were 10 cases of cerebral infarction, 9 cases of multiple lumen infarction, 8 cases of lacunar infarction, 4 cases of cerebral hemorrhage, 5 cases of cerebral thrombosis, and 7 cases of subarachnoid hemorrhage, while group B was marked with 8 cases of cerebral infarction, 13 cases of multiple lumen infarction, 9 cases of lacunar infarction, 4 cases of cerebral hemorrhage, 6 cases of cerebral thrombosis, and 4 cases of subarachnoid hemorrhage. Group C was comprised of 21 cases of cerebral infarction, 13 cases of multiple lumen infarction, 10 cases of lacunar infarction, 6 cases of cerebral hemorrhage, 5 cases of cerebral thrombosis, and 8 cases of subarachnoid hemorrhage. There were insignificant differences in the general data of each group (*P* > 0.05), with the comparability.

### 4.2. Algorithm Performance Tests

Figure 2(a) shows the comparison result of the three-layer threshold convergence performance, and Figure 2(b) shows that of the five-layer threshold convergence performance. MPSO tended to be a constant with the increase of iteration times. At the beginning of the iteration, the MPSO convergence rate was relatively slow, which also indicated that MPSO could not only search for the optimal threshold in a large range but also hold down to avoid premature convergence. Hence, the MPSO algorithm was superior to the other three algorithms in the test of convergence performance.

### 4.3. Comparison of Time Complexity of the Proposed Algorithm

The time complexity of different segmentation levels was compared in images of different sizes, and the 2nd/3rd/4th/5th levels were selected for comparative analysis. In Figure 3, as the number of image segmentation levels increased, the computation time increased little. Besides, as the image size increased, the corresponding time complexity also increased.  Figure 3(a) shows the image with 537 × 358 size which has the highest time complexity as compared to Figure 3(b) which shows the image with 321 × 481 size, and Figure 3(c) shows the image with 256 × 256 size. So, size reduction could be the one possible way of reducing the time complexity.

### 4.4. Comparison of CT Images

After the algorithm, CT images could reflect the anatomical details of different patients' brain CT manifestations as well as the infarction and the location of the lesion. The lesion was well segmented after the algorithm. In Figure 4, the orange area in the image represented the location of the lesion, and the red area represented the segmented part.

### 4.5. Comparison of Efficacy

In Table 3, there were 2 cases of cure, 4 cases of marked effectiveness, 5 cases of improvement, and 39 cases of ineffectiveness in group A. In group B, there were 6 cases of cure, 7 cases of marked effectiveness, 15 of improvement, and 22 cases of ineffectiveness. In group C, there were 17 cases of cure, 28 cases of marked effectiveness, 4 cases of improvement, and 1 case of ineffectiveness. The above statistics confirmed that patients in group C show a high rate of effectiveness as compared to the other two groups proving that anisodamine combined with chlorpromazine is the best remedy for intractable hiccups. The total efficiency was 98% in group C, 56% in group B, and 22% in group A (Figure 5). The total efficiency of group C was significantly different from that of group A and group B (*P* < 0.05).

### 4.6. Comparison of Satisfaction

A satisfaction of patients is the ultimate scale to measure the effectiveness of any treatment process (Table 4). 0 shows the statistics of various patients in different groups. 1 patient was satisfied, and 49 patients were dissatisfied in group A. In group B, 6 patients were very satisfied, 25 were satisfied, and 19 were dissatisfied. In group C, 29 patients were very satisfied, 18 were satisfied, and 3 were dissatisfied. The satisfaction rate was 94% in group C, 62% in group B, and 2% in group A (Figure 6). The total satisfaction of group C was significantly different from that of group A and group B (*P* < 0.05).

The histogram in Figure 6 confirmed that patients in group C were mostly satisfied with their treatment as compared to the other two groups, especially group A. The satisfaction of patients is a big achievement in any treatment process so the results clearly confirmed that anisodamine combined with chlorpromazine is the best treatment for intractable hiccups with the highest satisfaction rate in patients.

## 5. Discussion

A hiccup is also known as a diaphragm spasm which is caused by gastrointestinal dysfunction and stomach qi on the inverse moving diaphragm. In traditional Chinese medicine, the hiccup is, one or both diaphragms have paroxysmal involuntary contracture movement, with different duration. The main reflex center of a hiccup is in the 3rd to 5th cervical medullary segment with the vagus nerve being the afferent nerve, and the phrenic nerve is the efferent nerve [25, 26]. Central nervous system diseases, especially brainstem lesions, are easy to cause hiccups. In a very early period, people used acupoint stimulation to treat hiccups. After stimulation, stomach qi was reduced, and diaphragm spasm was relieved [27]. Zusanli is the acupoint of the foot yang stomach meridian, which has the function of regulating the spleen and stomach and depressing qi. Chlorpromazine can inhibit the central regulatory site of hiccup, delay the chemoreception of vomiting in the brain, block the ascending activation system of the brainstem reticular structure, and inhibit the excitation of the diaphragm. After the injection of drugs at the acupoint, acupuncture and drug effects are diffused through the nerve, and the reflex causes the inhibition of the cortical lesions induced electricity around the area, with long drug stagnation time in the acupoint. Moreover, the therapeutic effect is increased, and the intractable hiccup can be eliminated. A small dose of chlorpromazine injection can not only cause antiemetic effects in patients but also cause drowsiness if patients have a drug allergy. Anisodamine is an M-receptor blocker, which can relax the smooth muscle, relieve the smooth muscle spasm, and theoretically reduce hiccups [28]. Anisodamine combined with chlorpromazine was used to inject at the acupoint, and the drug efficacy was compared in the three groups. The total efficiency of anisodamine combined with chlorpromazine reached 98% marked by a 94% satisfaction rate, which was significantly different from the other two groups (*P* < 0.05). Gallagher [29] used a diaphragmatic drive band in the research of patients with an intractable hiccup in ischemic stroke, and the results showed that it could reduce the severity of hiccups in patients with ischemic stroke. Zhang and Gong [30] discussed the conditions of two patients with hiccups. A 46-year-old patient who had a 7-year history of intractable hiccups, with symptoms of dyspnea, dreaminess, fear of cold, and hypohidrosis, was diagnosed as an intractable or persistent hiccup. The acupuncture had no obvious effect on the treatment of this patient. In this work, there was also a patient who had intractable hiccup for 5 years. After drug treatment, it showed good results.

With the further development of image segmentation technology, many segmentation methods are using key measurement parameters to obtain the optimal segmentation threshold based on the principle of the optimal value of the objective function. In practical adoption, the amount of complex image data is quite large, so the processing time is relatively long. An intelligent optimization algorithm helps promote the development of image segmentation technology, which plays a crucial role in improving the image segmentation treatment and the segmentation speed [31, 32]. The intelligent optimization algorithm makes up for the shortcomings of a large amount of data and the slow calculation speed in image segmentation [33]. The calculation process of the threshold segmentation algorithm is simple, and the effect is good. Therefore, it develops rapidly in the segmentation technology. Different intelligent algorithms have been fully used in CT image segmentation. In this experiment, for the brain CT imaging of patients, the intelligent algorithm was used, which was helpful to improve the clarity of the images. The time complexity of different segmentation levels was compared in images of different sizes, and the 2nd/3rd/4th/5th levels were selected for the comparative analysis. With the increase in the number of image segmentation levels, the computation time increased little. Furthermore, the time complexity also increased with the increase of the image size. PSO algorithm was used to calculate the image characteristics. The complexity of image threshold segmentation was reduced. The improved algorithm could greatly improve the time complexity of multilayer image segmentation. The convergence performance of the improved algorithm was tested. The efficiency of the segmentation results and time consumption proposed in this work were verified.

## 6. Conclusion

CT diagnosis of patients with intractable hiccup after stroke was performed. When patients underwent CT examination, an intelligent algorithm was used to segment the images. Moreover, an unsupervised multilayer image threshold segmentation algorithm was obtained by using the 2D K-L divergence and the improved PSO algorithm, thus obtaining the clear CT images. Acupoint injection of anisodamine combined with chlorpromazine had better efficacy than the injection of anisodamine for intractable hiccup after stroke, with high safety and clinical promotion value. In this experiment, the problem of class imbalance in the segmentation network in image semantic segmentation needs to be further discussed. For the multilayer image segmentation, if the number of layers is automatically segmented, the consistency of image segmentation can be improved.

## Figures and Tables

**Figure 1:** Flow diagram of the algorithm.

**Figure 2:** The comparison results of the MPSO algorithm convergence performance.

**Figure 3:** Time complexity comparison of the MPSO algorithm.

**Figure 4:** Brain CT images.

**Figure 5:** Comparison of total efficiency among the three groups. Note: ∗ meant that the differences were considerable.

**Figure 6:** Comparison of satisfaction among the three groups. Note: ∗ meant that the differences were considerable.

**Algorithm 1:** Pseudocode of the MPSO algorithm.

**Table 1:** Evaluation criteria of efficacy.

Effect	Symptoms
Cure	After 1-2 treatments, the hiccups disappeared, and there was no recurrence after stopping the treatment.
Marked effectiveness	After 1-2 treatments, the hiccup disappeared, and the 6 h recurrence was effective again after treatment.
Improvement	After 1-2 times of treatment, the hiccup was relieved, but it did not disappear after retreatment.
Ineffectiveness	After 1-2 treatments, the hiccups were not relieved, and it did not disappear or it was even aggravated.

**Table 2:** Comparison of general data among the three groups.

Indexes	Group A (*n* = 50)	Group B (*n* = 50)	Group C (*n* = 50)
Female	31	26	29
Male	19	24	21
Cerebral infarction	10	8	21
Multiple lumen infarction	9	13	13
Lacunar infarction	8	9	10
Cerebral hemorrhage	4	4	6
Cerebral thrombosis	5	6	5
Subarachnoid Haemorrhage	7	4	8

**Table 3:** Comparison of evaluation of efficacy.

Group	Number	Cure	Marked effectiveness	Improvement	Ineffectiveness
Group A	50	2	4	5	39
Group B	50	6	7	15	22
Group C	50	17	28	4	1

**Table 4:** Comparison of satisfaction.

Group	Number	Very satisfied	Satisfied	Dissatisfied
Group A	50	0	1	49
Group B	50	6	25	19
Group C	50	29	18	3

## Data Availability

The datasets supporting the findings of this study are indicated in the article. Data will be made available on reasonable request.
